# Difficulties faced by university students with self-reported symptoms of attention-deficit hyperactivity disorder: a qualitative study

**DOI:** 10.1186/s13034-018-0218-3

**Published:** 2018-02-01

**Authors:** Soo Jin Kwon, Yoonjung Kim, Yeunhee Kwak

**Affiliations:** 1 Nursing Science Research Institute, Chung-Ang University, Seoul, Republic of Korea; 2 Faculty of Red Cross College of Nursing, Chung-Ang University, 84 Heukseok-Ro, Dongjack-Gu, Seoul, 156-756 Republic of Korea

**Keywords:** Attention-deficit hyperactivity disorder, Experience, Qualitative study, University students

## Abstract

**Background:**

Attention-deficit hyperactivity disorder (ADHD) persists into adolescence and adulthood; however, few studies have analyzed the experiences of university students with ADHD. This study explored the difficulties experienced by university students with ADHD symptoms.

**Methods:**

Between December 2015 and February 2016, face-to-face interviews were conducted with 12 university students with self-reported ADHD symptoms. Data were analyzed using thematic analysis.

**Results:**

Difficulties in university life were classified into four main themes (lack of daily routine, unsatisfactory academic performance and achievement, reduced interpersonal skills, and continuing worries) and analyzed. University students with ADHD symptoms had difficulties coping with repeated cycles of negative thoughts and worries, irregular lifestyles due to poor time management, dissatisfaction with academic performance and interpersonal relationships, self-dissatisfaction, and decreased self-esteem.

**Conclusion:**

To improve their university experience, students with ADHD should receive education about ways to stop worrying, to express emotions healthily, and to manage time efficiently.

## Background

Attention-deficit hyperactivity disorder (ADHD) has as its major symptoms inattention, impulsivity, and hyperactivity [1]. The prevalence rates of ADHD have been increasing over the past decades [2]. The revised Diagnostic and Statistical Manual of Mental Disorders (DSM-5) includes diagnostic criteria for adult ADHD, which differ from those for childhood ADHD [1]. The DSM-5 includes more developmentally expansive criteria and is expected to have a marked impact on the diagnosis and treatment of adult ADHD. A cross-national study of 11,422 adults in the United States and Europe reported that the prevalence of adult ADHD was approximately 3.4% and was significantly higher in higher-income than in lower-income countries (4.2% vs. 1.9%, respectively) [3]. Approximately 2–8% of university students have clinically significant ADHD symptoms [4]. Furthermore, studies in South Korea found that approximately 1.1% of adults had significant ADHD symptoms [5], and 7.6% of university students had ADHD [6].

Adults with ADHD have a lower quality of life than those without ADHD [7]. Similarly, college students with ADHD have a lower quality of life than do students without ADHD [8]; they have been shown to be more depressed and anxious, to be more easily angered or to suppress emotion, to have achieve less academically, and to be poorly supported in their relationships with their friends [9, 10]. ADHD symptoms have a negative impact on many aspects of life, including self-esteem, academic functioning, social functioning, and parent–child relationships [8, 11, 12]. Adults with ADHD are vulnerable to addiction; ADHD is often accompanied by addictive disorders [13] that are closely associated with sleep problems, leading to impairment in daily life [14].

In addition, adults with ADHD may experience frustration, depression, anxiety, difficulty in controlling emotions, interpersonal problems, and, in severe cases, personality disorders. They may often receive negative feedback from those around them and may exhibit suicidal behavior in response to repeated failures [4, 9, 10, 15–18]. Attending university is a particularly important period that affects future careers and overall social life; it is particularly challenging because of the adjustment to the new, unstructured environment that university students must make [19]. University students with ADHD experience a variety of academic, psychological, social, and mental problems [20]. Since university students with ADHD tend to have reduced life satisfaction and greater subjective pain than those without ADHD [21], there is a great need for ADHD treatment and interventions that support this vulnerable student cohort.

Although studies have been conducted to identify the support needs of university students with ADHD [18, 20], most of this research has focused on the experiences of students living in the United States, with little attention paid to diverse ethnic groups. To date, only a few studies have been conducted in Asia, making it difficult to generalize the findings to cross-national populations. The particular cultural demands faced by Korean university students, including the pressure to find a job and high parental expectations, may lead to difficulties such as mental health-related and self-centered behavioral problems [22, 23]. Given the low number of adults diagnosed with ADHD in Korea, the scarcity of related studies, and limited information about adult ADHD among the Korean population [10, 24], multifaceted studies and clinical approaches are needed to help Korean university students who have ADHD symptoms. To adequately address and evaluate the difficulties that such students experience, the condition must be explored from their perspective. Therefore, the present study aimed to investigate the difficulties experienced by Korean university students with ADHD symptoms so as to provide the basic data needed to develop appropriate interventions.

## Methods

### Study design

Data were collected by conducting in-depth, individual interviews with university students with ADHD symptoms, and were analyzed using thematic analysis.

### Participants

University students were recruited via an announcement posted on university bulletin boards. After signing the participation consent form, all volunteers were screened using the Korean version of the World Health Organization Adult ADHD Self-Report Scale (ASRS-v1.1) Symptom Checklist [25, 26]. Interviews were conducted with participants whose reported symptoms met more than four of the ASRS-v1.1 evaluation criteria [27]. A total of 12 participants (five men and seven women) were recruited, with a mean age of 22.2 years (range 20–29 years). Of these, two participants had been diagnosed with ADHD but were not receiving treatment at the time of the study; one participant had taken ADHD medication for approximately 2 years but had stopped taking it 3 years prior to enrolling in the study; the other participant was diagnosed with ADHD 8 years prior to enrolling in the study, had undergone counseling on four occasions, but had not received further treatment thereafter (Table 1).

**Table 1:** Participant demographic data (N = 12)

Number	Sex	Current age (years)	Current university year	Physician-diagnosed ADHD	Past medication
1	M	22	3	No	No
2	M	20	2	No	No
3	M	21	2	No	No
4	M	22	3	No	No
5	F	24	3	Yes	Yes
6	F	21	2	No	No
7	F	24	3	No	No
8	F	21	2	No	No
9	F	20	1	No	No
10	F	20	1	No	No
11	F	22	4	No	No
12	M	29	1	Yes	No

*ADHD* attention-deficit hyperactivity disorder

### Data collection

Data were collected between December 2015 and February 2016. Interviews with individual participants were held at a venue of the participant’s choice (the researcher’s office or an empty classroom). The ASRS-v1.1 took approximately 5–10 min to complete and each interview lasted 60–100 min. The interview questions were semi-structured. The key question was “What difficulties do you experience with your ADHD symptoms?” Additional questions included the following: (a) How are you doing currently? (b) How do you deal with the difficulties associated with ADHD symptoms? (c) How do you think ADHD symptoms are going to affect your future? (d) Which aspects of your ADHD symptoms do you wish to improve? and (e) Do you have additional thoughts or information you would like to share with us? The participants were encouraged to describe their experiences fully and the interviews were recorded. Participants’ nonverbal reactions and matters of importance, as determined by the interviewer, were written as comments in the filed notes. The recorded interviews were transcribed and analyzed.

### Data analysis

The collected data were analyzed using thematic analysis, as described by Braun and Clark [28]. This six-phase method focuses on identifying and analyzing the meanings of common themes. In the present study, phase 1 involved familiarization with the data. Meaningful information on participant experiences and difficulties in relation to their ADHD symptoms were identified by repeated reading of the transcribed data. In phase 2, initial codes were generated from the data. A total of 155 meaningful descriptions were extracted and coded. In phase 3, we searched for themes within the data. The codes were compared with candidate themes, and all data regarding candidate themes were collected. Overall, 27 candidate themes were extracted. In Phase 4, the themes were reviewed, and the researcher verified whether the extracted themes fitted in with the overall data. In total, four themes and nine subthemes were extracted. In phase 5, these themes and subthemes were defined and named, and, in Phase 6, the content was checked and the results described in a report.

To ensure the trustworthiness of this qualitative research, the present study considered the paradigms of research credibility, transferability, dependability, and confirmability set forth by Lincoln and Guba [29]. The study was conducted in accordance with qualitative research procedures and attempted to exclude biases and maintain neutrality throughout the study period. Extracted themes and subthemes were confirmed with two participants. Data analysis and result extractions were performed in collaboration with a professor of nursing science who has experience in qualitative research.

## Results

### Theme 1. Lack of a daily routine

Each of the participants in this study lacked a daily routine, which manifested as having an irregular lifestyle and consistently breaking promises to themselves and others. Furthermore, it was noted that the difference between the strict high school environment of the Korean education system and the more lenient university setting disconcerted participants.

#### Having an irregular lifestyle

The participants reported that during high school, their daily lives were regulated by their parents and teachers; however, at university, there was an increase in individual freedom and their daily lives became less structured. For example, they had irregular sleeping and eating patterns, with periods of binge eating and excessive drinking. As a result of their unsettled lives, the participants felt that they were wasting their time and were failing to achieve their desired goals and stability. The participants also reported that during the first and second years of university, they did whatever they wanted to do and did not experience any instability-related problems. The participants did not begin to experience difficulties in daily life until later in their university career, at which point they tried to change their lifestyles, but failed. The following is an excerpt from one of the participants:

I used to be good at cleaning the house and did all my own cooking, but it did not last long. Now, I wake up in the afternoon and fall asleep when the sun rises. My life is very erratic (Participant 4).

#### Plans not followed through

During their university careers, the participants made numerous attempts to learn new things or make plans to ensure regularity within their everyday lives, but they often gave up or failed to follow through on their intentions. Most of the participants received allowances from their families, but spent all their money on gifts for themselves or their friends. The participants would be embarrassed and reprimanded by their parents for failing to adhere to credit card limits. They recognized the need to change and enrolled in related support programs; however, they were repeatedly unable to alter their behavior and felt dejected. The following quotes are from two participants: “The funny thing is that I plan well but don’t put in the work. Even when I do start, I don’t finish as I intended to” (Participant 2) and “Since starting university, it seems that I am getting more and more haphazard. I think that the increasing amount of study I need to do is more than I can cope with and so it’s becoming pointless to plan” (Participant 11).

### Theme 2. Unsatisfactory academic performance and achievement

The participants expressed dissatisfaction with their academic performance and achievement. Despite acknowledging their student duty to complete assignments and to study, they lacked motivation. Many of the participants procrastinated, resulting in unsatisfactory outcomes. In addition, there was great variability in participant concentration levels for activities such as classes, which require maintained interest.

#### Procrastination

The participants were aware that they had to prepare for assignments or examinations in advance, yet they often procrastinated. Even if they started an assignment well in advance of a deadline, they could not concentrate properly on the task. The participants often stayed up all night before an examination or assignment deadline, or resorted to only studying on the day of the examination. By procrastinating, the participants failed to leave enough time for assignment revisions but, reportedly, could concentrate more easily under time pressure. The following is an excerpt from one of the interviews:

I vaguely think that I should start to work hard for this assignment after a certain time point because the assignment is due. When the time comes, I slowly start to work, but even if I sit down in the morning, I only get started in the evening (Participant 4).

#### Difficulty prioritizing and completing tasks

When presented with multiple tasks to complete, the participants stated that they did not know which task to complete first and experienced difficulty in completing tasks efficiently. Participants found it difficult to complete tasks because they were trying to focus on multiple subjects and several individual and group assignments. Further, when working in a group setting, the participants often put in extra effort to avoid upsetting their peers, but their peers often had to revise their work because of its poor quality. Overall, since the participants did not start assignments on time and had to finish them hastily, completion rates, results, and grades were poor. The following excerpts are from two of the participants:

I’ve been involved in a lot of activities. Because of this, there have been a lot of things that I haven’t been able to handle. I did try to study, but it didn’t work out well. So, I’ve just done extracurricular activities. I have a lot of regrets right now … The credits were very important for getting a job. It seems that I have never done my best in any assignment (Participant 5).

and “I feel like the pressure is getting so strong that I want to get it done anyhow, and fast. So, I don’t think I can do anything properly now. I often think, ‘Oh, why am I doing this?’” (Participant 6).

#### Interest-based participation

The students stated that they could only participate in campus activities, including classes, if activities were of interest to them. They stated that if they were taking an uninteresting class, they would be unable to focus and would instead waste time using their cell phones, scribbling, taking bathroom breaks, drinking beverages, or eating meals. The following excerpts are from two students: “I cannot keep still in a boring class. I intentionally don’t participate in it. It’s a waste of time. There are some professors who have interesting classes. I can take those classes” (Participant 11) and “If I listen [in a class] for about 10 min, I get more and more absent-minded. I stare at my watch, go to the bathroom although I do not want to go there, and play with my cell phone” (Participant 2).

### Theme 3. Unskilled interpersonal relationships

The participants stated that they had experienced difficulties building and maintaining interpersonal relationships since childhood. Throughout their lives, they stated that they had suppressed their negative emotions, practiced avoidance, and displayed extreme reactions (such as sudden emotional outbursts) within their relationships. The participants reported that their daily university lives were not disrupted by their interpersonal relationships; however, they were aware that this could be problematic when they started working after graduation.

#### Extreme reactions

The participants expressed extremely negative emotions when they experienced difficult situations within interpersonal relationships. Some participants reacted by avoiding a certain situation or person, and by hiding negative emotions during conflicts. In general, participants avoided expressing negative emotions to others and were angry with their families for making them fearful of expressing their negative emotions. Participants reported that their relationships often deteriorated if they expressed negative emotions; therefore, they avoided people they did not like and kept silent when in their company. Yet, some participants reacted by having a sudden emotional outburst, including episodes of excitement, screaming, and anger. The following two excerpts are from study participants: “I don’t want to see anyone I do not like, and because I don’t want to face these situations, I just don’t.” (Participant 7) and.

I don’t seem to be able to control my facial expression, although I can be patient in front of people. Sometimes I get angry at my friends or family, and I apologize to them afterwards when I feel relaxed or calm (Participant 3).

#### Difficulty building and maintaining relationships

Participants tried to overcome difficulties within interpersonal relationships by convincing themselves that they were fine with others or that their relationships were improving. However, failure to resolve conflicts within these relationships caused the participants to have difficulties developing deeper relationships with other people. Specifically, participants often encountered conflicts in relation to being late or absent for appointments. Further, the participants stated that their friends understood that they could occasionally not keep appointment times. Unlike high school, university affords students the opportunity to choose their own classes and make their own schedules; therefore, they have more freedom to live their lives without maintaining close relationships with other people. As a result, students often remain isolated and only interact with a small group of peers when necessary. The participants expressed difficulty in adjusting to certain subjects that required interactions with other people, with some participants even wanting to switch to subjects requiring fewer interpersonal relationships. The following quote is from one of the participants: “Interpersonal relationships were the most challenging for me. My biggest worry is always interpersonal relationships. I have always found maintaining deeper and longer relationships with others difficult” (Participant 6).

### Theme 4. Continuous worry

Although the participants occasionally acted impulsively, they were generally introspective in their daily lives, and these thoughts caused worry. The participants tended to brood over past events and worried about things that had not happened yet. Furthermore, because of bad past experiences, the participants did not trust themselves in the future, thereby increasing their anxiety.

#### Obsession with past events

The participants tended to repeatedly think about and regret past events. Participants stated that if past events were associated with negative thoughts, then they often engaged in a perpetual cycle of worry. However, they did recognize that it was unnecessary to keep thinking about the past and that it was not important to their current situation. The participants were mostly preoccupied with thoughts revolving around everyday matters, such as whether they satisfactorily submitted an examination paper, submitted their assignments without errors, closed the door properly, or whether or not there were problems in their relationships with other people. The following are excerpts from two participants: “I’m worried even though I think ‘Oh, stop worrying. It’s already over.’” (Participant 5) and “I am afraid I have a lot of worries about relationships with other people. When someone else does something wrong to me, I quickly forget it. However, when I do something wrong, I keep on remembering it” (Participant 9).

#### Self-distrust

The participants underestimated themselves because of negative past experiences. When they obsessed about past events, they often experienced anxiety and worry about the future. Specifically, the participants were concerned about finding professional fields or jobs that would be suitable for their perceived weaknesses. Participants expressed a desire to obtain an interesting job that would allow them to work independently, rather than collectively. However, the content of their future job was not concrete or realistic. Below are two interview excerpts: “I am afraid that overall, I fall short. If the average score of ordinary people is 50, I feel like I will score 40. Overall, I think I am a bit lacking in ability compared to other people” (Participant 3) and “I worry a lot about making mistakes. For example, I keep worrying that my answer sheet will not be properly submitted when I take an exam” (Participant 7).

## Discussion

The present study aimed to analyze the difficulties experienced by university students with ADHD symptoms. A total of 12 eligible students were interviewed and four themes emerged during the analysis. The first theme was lack of a daily routine. University students with ADHD symptoms did not implement their plans well because of their inattention, impulsivity, and the lack of regularity within their daily lives. Hyperactivity, which is common in pediatric patients with ADHD, decreases markedly with age, such that superficial activity is maintained at a relatively reasonable level in adult patients with ADHD [30]. However, the present study shows that certain ADHD-related difficulties persist into adulthood, including impulsivity, inattention, difficulty in controlling emotions, and inability to systematize [15, 18]. In addition, previous studies have indicated that university students with ADHD symptoms have irregular sleeping hours and lower sleep quality [18, 31], and eat irregular meals or occasionally partake in binge eating [31, 32]. These observations are consistent with the results of the present study. Many studies have shown that university students with an ADHD tendency or diagnosis have more difficulties with alcohol, smoking, and internet and smartphone addiction than do other students [6, 22, 26, 33, 34]. These outcomes further support the theory that university students with ADHD symptoms lack structure in their daily lives. Therefore, attention, support, and other appropriate interventions would help these students manage their daily life schedule, including their sleeping and eating behaviors, while coaching programs or organizational skills intervention programs may help them manage their time more efficiently [35, 36].

The second theme was unsatisfactory academic performance and achievement. Even if the students made plans to study in advance, they failed to prioritize and complete tasks. This resulted in unsatisfactory academic performance and achievement. The students made efforts to overcome these problems, but their concentration waned with lack of interest, and they struggled with repeated failures. Previous studies have reported that such students have difficulty planning and completing tasks as a result of procrastination or indecision, and thus do not manage their time well [37, 38]. Other studies have reported that university students with ADHD symptoms have low academic performance as a result of difficulties with concentrating on their studies and completing assignments, worries about studying and having high test anxiety, and not applying appropriate learning strategies, which all lead to problems with adjusting to university life [4, 9, 16–18, 21, 39]. Such difficulties in adjusting to university life can extend to difficulties in social functioning in adulthood. For example, these students may fail to secure employment or may find only low income employment [3, 40]. Therefore, programs promoting academic strategies and time management skills should be implemented to help these students improve their academic performance and educational achievements. As in previous studies, working memory training or self-monitoring can be applied to support their learning [41, 42]. In addition, our results indicate that these students should be encouraged to concentrate on their areas of interest, as this strategy might help them to better select and adapt to their future jobs.

The third theme was unskilled interpersonal relationships. The participants reported having extreme reactions in interpersonal relationships and experienced difficulties in forming and maintaining relationships as a result of this impulsivity. Previous studies have shown that university students with ADHD have higher levels of anger and greater difficulty in controlling emotions than their peers; therefore, these students often express anger in socially unacceptable ways [10, 33]. Furthermore, studies have reported that university students with ADHD tend to be more aggressive or confrontational in stressful situations than their peers; therefore, they often experience difficulties in forming relationships with other people [4, 10]. Since ADHD is associated with certain characteristics, such as inattentiveness and impulsivity, individuals diagnosed with ADHD tend not to pay enough attention to the feelings and desires of others, often interfering in a criticizing and controlling way, and causing conflict, disappointment, and distrust [10]. Research indicates that anger and aggressiveness negatively impact interpersonal relationships [43]. The establishment of self-identity and formation of personal relationships are important developmental tasks for university students. The lack of social skills in patients with ADHD is already known, but until now, the mechanisms leading to such difficulties have remained obscure; this study provides an understanding of why social skills are lacking. Impaired interpersonal competence can cause serious psychological maladjustment and low self-esteem, which have serious effects on life satisfaction [21]. It is, thus, important for college students with ADHD to be educated about how to express their negative feelings more healthily (rather than expressing extreme anger or displaying avoidance), to learn interpersonal skills, and to consider the effects that their ADHD symptoms can have on their relationships with others.

The final theme was continuous worry. This study found that although university students with ADHD symptoms tried to overcome these tendencies, they had high levels of self-distrust as a result of perpetually repeating cycles involving obsessing over past events and worrying about future failures. This can reduce their expectations for the future, gradually exacerbating their negative functioning. Previous studies have reported that university students with ADHD tendencies demonstrate a poorer adjustment to university life, exhibiting higher rates of depression and anxiety and lower than usual self-esteem and self-efficacy [6, 10, 21, 30, 44]. Patients with ADHD are known to have very poor tolerance for stress and dysfunctional coping styles [45]. As they are often inefficient and have difficulty adjusting to major life obligations, such as academic studies or occupations, these individuals are more likely than the general population to experience stress-causing negative life events [46, 47]. They may be very worried about repeated failures, the negative feedback they receive as a result of low academic performance, and interpersonal difficulties. These students are also more easily distracted. Time management is very important for enhancing self-efficacy and academic performance among university students [19]. Therefore, students should be taught effective time management skills to help them perform tasks efficiently and achieve a good work-life balance.

The final theme, the extent to which these students constantly worry about past mistakes and potential future ones, is important in this study. As a result of their history of repeated negative experiences and failed efforts, they come to distrust themselves and their ability to achieve their goals, which leads to further demoralization, loss of motivation, and progressive worsening of their functioning over time. Therefore, when providing interventions, it is necessary to repeatedly reduce negative feedback and to reinforce positive motivation for the future; this is an important implication arising from this study.

In summary, university students with ADHD symptoms have difficulties coping with repeated cycles of negative thoughts and worries, irregular lifestyles as a result of poor time management, dissatisfaction with academic performance and interpersonal relationships, and self-dissatisfaction. Although individual or group cognitive-behavioral therapy, mindfulness training, and coaching [20], may be helpful, it is necessary to consider the social and cultural environment of the subject based on the results of this study when applying and developing programs appropriate for them. To help these students live a healthy lifestyle at university, they should be properly diagnosed and educated about ADHD, how to prevent worrying, how to express emotions healthily, and how to effectively manage time. Social awareness of adult ADHD should also be enhanced.

This study has several limitations. First, the subjects were Korean university students; therefore, caution must be applied when generalizing these results to adults from other countries, cultures, and age groups. Further studies of university students or adults from different populations are needed. Second, participants were selected on the basis of self-reported ADHD symptoms; the experiences of and findings related to those formally diagnosed with ADHD or receiving ADHD treatment may differ. The findings of this study need to be captured and quantified using standardized rating instruments, and replicated in larger samples with fully diagnosed students. Despite these limitations, we believe that this study is important because it is the first to analyze difficulties from the perspective of Korean university students with ADHD symptoms. In addition, this study highlights the importance of developing intervention programs for such university students.

## Conclusions

When the difficulties experienced by Korean university students with ADHD symptoms were analyzed, four main themes were identified, including lack of a regular daily routine, unsatisfactory academic performance and achievement, unskilled interpersonal relationships, and an ongoing tendency to worry. Students were aware of these difficulties and tried to overcome them by self-discipline. However, their self-esteem was lowered as a result of repeated cycles of inattentiveness and impulsivity. Therefore, to improve their experiences, university students with ADHD symptoms must develop insight into their diagnosis and be educated about ways to stop worrying and to effectively manage time. It is also important for universities to provide students with access to resources for life management.

## Abbreviations

ADHD: attention-deficit hyperactivity disorder
DSM: diagnostic and statistical manual of mental disorders
ASRS: Adult ADHD Self-Report Scale
